The article "The Expression of ephrinA1/ephA2 Receptor Increases in Chronic Rhinosinusitis and ephrinA1/ephA2 Signaling Affects Rhinovirus-Induced Innate Immunity in Human Sinonasal Epithelial Cells" was retracted in 2024. Reason: concerns about the images.

# The Expression of ephrinA1/ephA2 Receptor Increases in Chronic Rhinosinusitis and ephrinA1/ephA2 Signaling Affects Rhinovirus-Induced Innate Immunity in Human Sinonasal Epithelial Cells

**DOI:** 10.3389/fimmu.2021.793517

**Published:** 2021-12-16

**Authors:** Sang Hag Lee, Sung Hoon Kang, Mun Soo Han, Ji Won Kwak, Hyeon Geun Kim, Tae Hoon Lee, Da Bin Lee, Tae Hoon Kim

**Affiliations:** Department of Otorhinolaryngology-Head & Neck Surgery, College of Medicine, Korea University, Seoul, South Korea

**Keywords:** ephrinA1/ephA2 signaling, chronic rhinosinusitis with nasal polyps, chronic rhinosinusitis without nasal polyps, type I interferon, type III interferon, interferon stimulated genes, rhinovirus, innate immune response

## Abstract

EphA2 receptor and its ephrin ligands are involved in virus infection, epithelial permeability, and chemokine secretion. We hypothesized that ephrinA1/ephA2 signaling participates in rhinovirus (RV)-induced antiviral immune response in sinonasal mucosa of patients with chronic rhinosinusitis (CRS). Therefore, we investigated the expression of ephrinA1/ephA2 in normal and inflamed sinonasal mucosa and evaluated whether they regulate chemokine secretion and the production of antiviral immune mediators including interferons (IFNs) in RV-infected human primary sinonasal epithelial cells. For this purpose, the expression and distribution of ephrinA1/ephA2 in sinonasal mucosa were evaluated with RT-qPCR, immunofluorescence, and western blot. Their roles in chemokine secretion and the production of antiviral immune mediators such as type I and III IFNs, and interferon stimulated genes were evaluated by stimulating ephA2 with ephrinA1 and inactivating ephA2 with ephA2 siRNA or inhibitor in cells exposed to RV and poly(I:C). We found that ephrinA1/ephA2 were expressed in normal mucosa and their levels increased in inflamed sinonasal mucosa of CRS patients. RV infection or poly(I:C) treatment induced chemokine secretion which were attenuated by blocking the action of ephA2 with ephA2 siRNA or inhibitor. The production of antiviral immune mediators enhanced by rhinovirus or poly (I:C) is increased by blocking ephA2 compared with that of cells stimulated by either rhinovirus or poly(I:C) alone. In addition, blocking ephA2 attenuated RV replication in cultured cells. Taken together, these results describe a novel role of ephrinA1/ephA2 signaling in antiviral innate immune response in sinonasal epithelium, suggesting their participation in RV-induced development and exacerbations of CRS.

## Introduction

Chronic rhinosinusitis (CRS) is a heterogenous mucosal inflammation of the nasal cavity and paranasal sinuses (1). Although the pathophysiological causes of CRS remain unclear, accumulating evidence suggests that abnormal immune response of sinonasal mucosa to respiratory viral infection can progress to secondary bacterial infection and induce the exacerbation of CRS (2–6).

The article "The Expression of ephrinA1/ephA2 Receptor Increases in Chronic Rhinosinusitis and ephrinA1/ephA2 Signaling Affects Rhinovirus-Induced Innate Immunity in Human Sinonasal Epithelial Cells" was retracted in 2024. Reason: concerns about the images.

Rhinovirus (RV) infections are the most common cause of viral upper airway infections (4, 7, 8). However, it is unclear why they are self-limiting in the majority of persons, but in others can advance to bacterial sinusitis and enhance CRS exacerbations (2–6). A deeper understanding of host defense factors that contribute to effective protection against respiratory viral infection may aid in the prevention of disease progression and in the development of new therapeutic target.

RVs initially encounters sinonasal epithelial cells and impair epithelial barrier function by disrupting the junction proteins, including ZO-1 (9–11). During the early course of RV infection, pattern recognition receptors, such as Toll-Like receptor 3 (TLR3) expressed in superficial epithelial cells, are activated to produce anti-viral immune mediators such as type I and III interferon (IFN) to prevent the viral infection (12–14). Simultaneously, RV-infected epithelial cells produce chemokines which trigger the chemoattraction of immune cells into infection site to facilitate viral clearance (13, 14).

Numerous studies have demonstrated impaired antiviral innate immune responses toward RV infection in patients with asthma and COPD, which is an important cause of acute exacerbations (15–18). The expression of IFN-α and IFN-β in bronchial epithelium is deficient in patients with asthma and this epithelial deficiency is involved in viral load and clinical illness severity (19). Patients with COPD when clinically stable and during virus-associated exacerbation exhibit lower expression levels of type I and III IFNs (20). As observed in patients with asthma and COPD, patients with CRS showed lower expression levels of type I and III IFNs, and IFN-stimulated genes (ISGs), which suggests that their deficiency may impair the antiviral innate response (12). However, the specific mechanisms underlying deficient expression of anti-viral mediators by viral infection has not been well established.

An interesting group in this regard is the erythropoietin-producing human hepatocellular carcinoma (eph) receptor tyrosine kinases and their ligands ephrins (21). Based on ligand binding preferences, the ephrin receptor family are divided into two broad classes, ephA and ephB receptors, which are involved in various biological functions, such as cell assembly, migration, and adhesion (22). Specifically, ephrinA1 and ephA2 are recognized as key regulators of inflammation (23). More recently, ephA2 were reported to serve as the entry receptor for microbial organisms, participating in host-pathogens interaction. In oral epithelial cells and gastric mucosa, ephA2 recognizes *Candida albicans* and *Helicobacter pylori*, acting as a pattern recognition receptor and inducing adaptive protective host responses against these organisms (24, 25). Specifically, the ephA2 receptor was reported to function as a host cofactor for Kaposi’s sarcoma-associated herpesvirus (KSHV) and an entry receptor for Epstein-Barr virus (EBV) (26–28). Knockdown of ephA2 significantly reduced KSHV entry and EphA2 overexpression significantly increased EBV infection (26–28). An EBV-encoded early lytic protein, BERF1, inhibited the IFN-β production, disrupting the host innate immunity (29).

The article "The Expression of ephrinA1/ephA2 Receptor Increases in Chronic Rhinosinusitis and ephrinA1/ephA2 Signaling Affects Rhinovirus-Induced Innate Immunity in Human Sinonasal Epithelial Cells" was retracted in 2024. Reason: concerns about the images.

Previous studies have demonstrated that ephA2 deficiency attenuated pulmonary inflammation by decreasing inflammatory response and attenuating the secretion of inflammatory cytokines (30). Tobacco smoke exposure induces EphA2 expression and the inhibition of ephA2 expression blocked tobacco smoke-mediated epithelial permeability (31). Concentration in lung tissue of neutrophil and monocyte chemoattractants were markedly lower in ephA2-deficient mice, suggesting that ephA2 regulates inflammation (32). Stimulation of lung endothelial EphA2 receptors with ephrinA1 ligand altered pulmonary vascular permeability (33). EphA2 receptor was increased in viral infection, contributing to vascular leak in the injured lung (34). The ephrinA1/ephA2 signaling participates in the maintenance of the intestinal barrier to regulate the expression of adherens junction (35). However, there is no published description on the relationship between ephrinA1/ephA2 signaling pathways and RV infection in the sinonasal mucosa. Thus, we hypothesized that the ephrinA1/ephA2 signaling may attenuate the RV-induced antiviral immune response in CRS.

In the present study, we evaluated the role of the ephrinA1/ephA2 receptor in RV-induced antiviral innate immune responses such as chemokine production and the production of anti-viral immune mediators such as type I (IFN-β) and III IFNs (IFN-λ1 and IFN-λ2), and ISGs (viperin, Mx, and OAS). Furthermore, we evaluated whether cross-talk exists between the ephrinA1/ephA2 signaling and other known signaling pathways in RV-induced antiviral immune response.

## Materials and Methods

### Subjects and Sample Collection

A total of 134 patients were enrolled; 25 patients were controls, 36 patients had CRS without nasal polyps (CRSsNP), and 73 had CRS with nasal polyps (CRSwNP) (35 non-eosinophilic, 38; eosinophilic) (**Supplementary Table 1**). The patients were classified into CRSsNP or CRSwNP based on the diagnostic parameters outlined by the European Position Paper (1). Normal sinus mucosal sampling was conducted in the ethmoid sinus of patients with blowout fracture as a control and inflamed sinus mucosa was obtained from the ethmoid sinus of patients with CRS during surgery, respectively. The ethmoid sinus mucosal tissues obtained during surgery were frozen at -75°C for reverse transcriptase-quantitative PCR (RT-qPCR) and western blot analysis and were also prepared for culture of normal and inflammatory sinonasal epithelial cells. A part of samples was fixed in 4% paraformaldehyde for immunofluorescent and histologic analyses. CRSwNP was divided into eosinophilic or non-eosinophilic type by calculating the mean number of eosinophils as described previously (36).

The article "The Expression of ephrinA1/ephA2 Receptor Increases in Chronic Rhinosinusitis and ephrinA1/ephA2 Signaling Affects Rhinovirus-Induced Innate Immunity in Human Sinonasal Epithelial Cells" was retracted in 2024. Reason: concerns about the images.

The review board and ethics committee approved all experimental procedures, and written informed consent was obtained from all subjects. The radiographic and endoscopic severity scores of sinus disease, and symptom scores were assessed as described previously (**Supplementary Table 1**) (37–39). Subjects had no history of allergic rhinitis, asthma, previous sinus surgery, or viral URI and were excluded if they took medication, including steroids, antibiotics, or antihistamines 3 months before the endoscopic surgery. Symptoms of viral upper airway infection was determined based on the Jackson scale (40).

### Culture of Normal and Inflammatory Sinonasal Epithelial Cell

Normal and inflammatory ethmoid sinus mucosa obtained from endoscopic reduction in patients with blowout fracture and patients with CRSwNP and CRSsNP was used for culture of normal and inflammatory epithelial cells in the presents study as previously described (12). Ethmoid sinus mucosa obtained during surgery was digested with 0.5% dispase in Dulbecco’s modified Eagle’s medium (DMEM)/F12 (GenDEPOT, TX, USA). Thereafter, the epithelial cells were mechanically harvested from ethmoid sinus mucosa and were centrifuged at 1200 RPM for 3 min. Cells in submerged cultures were grown in six-well plates filled with Bronchial epithelial cell medium (BEpiCM; ScienCell, Carlsbad, CA, USA). Thereafter, 2 x 10^5^ cultured epithelial cells were cultured under air-liquid interface (ALI) in the SPLInsert system (polyethylene terephthalate, 0.4 μm, pore size, 6.5 mm, SPL, Pocheon City, Kyung Ki DO, Korea). Both sides of the SPLInsert were filled with BEGM : DMEM/F12 (Lonza Walkersville Inc., Walkersville, MD, USA) under submersion for the first 3 days. An ALI was created on day 4 by removing the apical medium and feeding the culture from the basal compartment. The culture medium was changed 3 time per week after initiation of ALI. All experiments were performed on cultured epithelial cells after the creation of ALI.

The article "The Expression of ephrinA1/ephA2 Receptor Increases in Chronic Rhinosinusitis and ephrinA1/ephA2 Signaling Affects Rhinovirus-Induced Innate Immunity in Human Sinonasal Epithelial Cells" was retracted in 2024. Reason: concerns about the images.

### RV Propagation and Infection

Human RV 16 (ATCC VR-283PQ) was propagated in H1HeLa cells (ATCC, Manassas, VA, USA) in T175 tissue culture flasks at 33°C/5% CO_2_ in Eagle’s minimum essential medium (ATCC). After the cytopathic effect of the infected cells exceeds 70%, the virus was purified from harvested cell suspension, according to ATCC recommendations.

To determine the virus titer, H1HeLa cells were cultured in 96-well tissue culture plates and infected with 10-fold serial dilutions of purified stock virus. Infected cells were evaluated daily for cytopathic effect by microscopic examination for 5 days, and viral titer was determined by tissue culture infectivity dose (TCID_50_) assay as described previously (41).

### Effect of TLR3 Agonist, RV Infection, and Type 1 and Type 2 Cytokines on Expression of EphrinA1 and EphA2 Receptor

**N**ormal human primary epithelial cells grown in ALI were stimulated with TLR3 agonist [poly(I:C), 10 ug/ml, *In vivo*Gene, CA, USA] and treated with Type 1 and Type 2 cytokines such as TNF-α, IFN-γ, IL-4, IL-5, and IL-13 (10 ng/mL, R&D systems, Minneapolis, MN) for 24 hours. Thereafter, the levels of ephrinA1, ephA2, and phosphorylated ephA2 were evaluated with RT-qPCR and western blot.

Normal and inflammatory human primary epithelial cells grown in ALI were apically inoculated with human RV 16 at a MOI of 1 viral particle per apically exposed epithelial cell and were incubated for 4 h in an incubator with 5% CO_2_ at 33°C. After aspirating nonattached virus, cultured cells were additionally incubated for 20 h at 33°C. This MOI was selected because we determined previously that MOI of 1 do not induce loss of cells. After 24 hours, ephrinA1, ephA2, and phosphorylated ephA2 levels were evaluated with RT-qPCR and western blot.

### Effect of EphrinA1/ephA2 Signaling Axis on the Production of Chemokines and Antiviral Immune Mediators Induced by Human RV 16 and TLR3 Agonist

To analyze whether the ephrinA1/ephA2 signaling may regulate the expression of chemokine and antiviral immune mediators enhanced by human RV 16 and poly (I:C), the cultured epithelial cells were transfected with ephA2 siRNA or pretreated with ephA2 inhibitor (1 μM, ALW-II-41-27, APExBIO, TX, USA) for 48 hours respectively. Thereafter, cultured cells were incubated with 1 MOI of RV 16, poly (I:C) at a concentration of 10 uM, or ephrin A1 (1, 10, 25, and 50 ng/ml, R&D systems, Minneapolis, MN). After 24 hours, cultured cells and supernatants were harvested to evaluate the expression levels of the following mediators; IL-8, IL-6, ENA78, MIP1-α, RANTES, MCP-1, type I (IFN-β) and type III (IFN-**λ)** interferons, and IFN-stimulated genes such as viperin, Mx, and OAS with RT-qPCR, western blot, and ELISA. Additionally, the expression of downstream signal transducers such as P13K/Akt/NF-κB pathways, and TBK/IKKϵ/interferon regulatory factor 3 (IRF3) pathways was evaluated with western blotting. Furthermore, additional experiments were conducted to investigate whether the inhibition of the TBK/IKKϵ/interferon regulatory factor 3 (IRF3) pathways has an effect on RV-and/or poly(I:C)-induced IFN and ISG expression using MRT67307 (TBK/IKKϵ inhibitor, *In vivo*Gen, CA, USA) and G140 (IRF inhibitor, *In vivo*Gen).

The article "The Expression of ephrinA1/ephA2 Receptor Increases in Chronic Rhinosinusitis and ephrinA1/ephA2 Signaling Affects Rhinovirus-Induced Innate Immunity in Human Sinonasal Epithelial Cells" was retracted in 2024. Reason: concerns about the images.

### Effects of ephA2 Receptor on the Rhinoviral Replication

To estimate the amount of viral infection that had occurred during the exposure period, medium and cells harvested at the end of the infection were stored at -75°C for the determination of viral content. To evaluate whether viral replication in cultured cells may be affected by blocking ephA2 receptor, the cultured epithelial cells were transfected with ephA2 siRNA or pretreated with ephA2 inhibitor (1 μM, ALW-II-41-27, APExBIO, TX, USA) for 48 hours respectively. Thereafter, cultured cells were incubated with 1 MOI of RV 16 and were harvested in hour: 6, 12, 24, and 48 after infection. Thereafter, viral RNA was isolated with the QIAamp Viral RNA Mini Kit (Qiagen, Ontario, CANADA) and subjected to RT-qPCR using the following primers and probe: forward primer; AGCCTGCGTGGCTGCC; reverse primer: ACACCCAAAGTAGTCGCTCCC; probe: TCCGGCCCCTGAAT.

### Transfection of Sinonasal Epithelial Cells with EphA2 siRNA

Cultured epithelial cells were transfected with ephA2 siRNA and scrambled siRNA as control using Lipofectamine 2000 (Invitrogen, Carlsbad, CA, USA) according to the manufacturer’s recommendations. Briefly, 75 pmole of the siRNA was diluted in 50 ul of Opti-MEM^®^ Medium and then mixed with another 50 ul of Opti-MEM^®^ Medium containing 3 ul of lipofectamine 2000 (Invitrogen). These transfection mixtures were added into each insert. Subsequently, 2 x 10^5^ cultured epithelial cells suspended in another 100 ul of Opti- MEM^®^ Medium were added into the same insert. The well plates containing these inserts were incubated at 37°C in a 5% CO2 incubator for 24 h. Thereafter, the Opti-MEM^®^ Medium on the apical surface of each insert was aspirated and replaced with Bronchial epithelial cell medium. Once the monolayer of cultured epithelial cells has reached 100% confluence on the inserts, Bronchial epithelial cell medium on the apical surface was aspirated and replaced with 100 ul of the Opti-MEM^®^ Medium containing 500 nmole/L of the siRNA mixed with Lipofectamine 2000 reagent again, and incubated for another 24 h at 37°C. Thereafter, transfection solution was then removed and replaced with ALI media. The plate was then incubated for 48 h or longer for transfection experiments.

The article "The Expression of ephrinA1/ephA2 Receptor Increases in Chronic Rhinosinusitis and ephrinA1/ephA2 Signaling Affects Rhinovirus-Induced Innate Immunity in Human Sinonasal Epithelial Cells" was retracted in 2024. Reason: concerns about the images.

EphA2 siRNA were synthesized as a purified duplex (Bioneer Co., Daejeon, Korea) and the sequences were as follows: AGUAGAGGUUGAAAGUCU (sense) and GAGACUUUCAACCUCUAC (antisense). The resultant genes and protein expression of ephA2 were determined by RT-qPCR and western blotting, respectively.

### Cell Viability

Cell viability was assessed using the MTT assay [3-(4,5-dimethylthiazol-2-yl)-2,5-diphenyltetrazolium bromide, Abcam, Cambridge, UK], as described previously (12).

### RT-qPCR, Western Blot, and Immunofluorescence

Total cellular RNA was extracted from mucosal tissues and cultured epithelial cells by using Qiazol lysis reagent (QIAZEN Inc, CA, USA) and was processed to the synthesis of. complementary DNA in a reaction mixture containing MML-V (Invitrogen) and oilgo (dT) primers (GenDEPOT, TX, USA). Gene expression levels were conducted using SYBR Premix EX Taq™ (Takara bio, Shiga, Japan). The mean threshold cycle (Ct) values were normalized to glyceraldehyde-3-phosphate dehydrogenase (GAPDH), and the relative mRNA levels of target genes were analyzed with 2^-ΔΔCt^. The primer sequences of each genes are listed in **Supplementary Table 2**.

For western blot, frozen mucosal tissues and cultured epithelial cells were disrupted in RIFA buffer (GenDEPOT). The BCA Protein Assay Kit (Bio-Rad, Bedford, MA, USA) was used to measure the protein content and equal amounts of proteins (50 ug) were separated on SDS-PAGE and transferred onto nitrocellulose membranes (Bio-Rad, Bedford, MA, USA). Thereafter, the membranes were blocked for 1 hour at room temperature with PBS-Tween 20 containing 5% skim milk and then incubated with primary antibodies such as anti-mouse-ephrinA1(A-5) antibody (sc-377362, 1:250. Santa Cruz Biotechnology), anti-rabbit-ephrinA2 antibody (ab-5386, 1: 250, Abcam), anti-rabbit-phospho-ephrinA2 antibody (D9A1) (#6347, 1:1000, Cell Signaling Technologies), anti-OAS antibody (ab272492, 1:500, Abcam), anti-goat-Mx antibody (AF7946, 1 ug/ml, R&D), anti-viperin antibody (G-8) (sc-390342, 1:250, Santa Cruz), anti-rabbit-PI3K antibody (C73F8) (#4249, 1:1000, Cell Signaling Technologies), anti-rabbit-phospho PI3K antibody (E3U1H) (#17366, 1:1000, Cell Signaling Technologies), anti-rabbit-Akt antibody (11E7) (#4685, 1:1000, Cell Signaling Technologies), anti-rabbit-phospho Akt antibody (D9E) (#4060, 1:2000, Cell Signaling Technologies), anti-rabbit-NF-κB antibody (D14E12) (#8242, 1:1000, Cell Signaling Technologies), anti-rabbit-phospho-NF-κB antibody (92H1) (#3033, 1:1000, Cell Signaling Technologies), anti-rabbit-TBK antibody (E813G) (#38066, 1:1000, Cell Signaling Technologies), anti-rabbit-phospho-TBK antibody (D52C2) (#5483, 1:1000, Cell Signaling Technologies), anti-rabbit-IKKϵ antibody (D61F9) (#3416, 1:1000, Cell Signaling Technologies), anti-rabbit-phospho-IKKϵ antibody (D1B7) (#8766, 1:1000, Cell Signaling Technologies), anti-rabbit-IRF3 antibody (D614C) (#11904, 1:1000, Cell Signaling Technologies), anti-rabbit-phospho-IRF3 antibody (E7J8G) (#37829, 1;1000, Cell Signaling Technologies) and anti-β-actin (C-2) (sc-8432, 1:200, Santa Cruz). Bands were detected with an ECL detection kit (Gendepot, Tx, USA). The intensity of each protein was normalized against that of the corresponding β-actin bands.

The article "The Expression of ephrinA1/ephA2 Receptor Increases in Chronic Rhinosinusitis and ephrinA1/ephA2 Signaling Affects Rhinovirus-Induced Innate Immunity in Human Sinonasal Epithelial Cells" was retracted in 2024. Reason: concerns about the images.

Tissue sections (14 µm) were processed for immunofluorescence, incubating with anti-mouse ephrinA1 (A-5) antibody (sc-377362, 1: 100, Santa Cruz) and anti-rabbit-ephrinA2 antibody (ab-5386, 1: 50, Abcam) overnight at 4°C. After washing, the sections were subsequently labeled with an Alexa 488 fluorescent dye-conjugated anti-mouse IgG and anti-rabbit IgG (Abcam), respectively. To verify the specificity of staining, adjacent sections were preincubated with the antigen to antibody mixture at a working dilution of 10:1 at 4 °C using blocking peptide (sc-377362 P) for ephrinA1 and ephrinA2 protein (ab114898) for ephrinA2.

### Determination of the Production of Chemokines, Type I (IFN- β), and Type III (IFN-λ) Interferons by ELISA

Levels of chemokines and antiviral immune mediators, including IL-8, IL-6, ENA78, MIP1-α, RANTES, MCP-1, type I (IFN- β) and type III IFN (IFN-λ1 and IFN-λ2), were measured in cell-free supernatants using commercial ELISA kits (R&D Systems), according to a manufacture’s recommendation.

### Statistical Analyses

Statistical analysis was performed using SPSS for Windows (version 16.0.0; SPSS, Chicago, IL, USA). Population normality and homogeneity of variance were evaluated for all data that were considered nonparametric. A Kruskal-Wallis test with a Dunn’s *post-hoc* test was conducted to compare demographics and clinical parameters of the four groups and the data from RT-qPCR, western blotting, and ELISA. Results are presented as median and range. P <0.05 was considered statistically significant.

## Results

The clinical characteristics of participants enrolled in this study are listed in **Supplementary Table 1**. The distribution of age and sex did not significantly differ among the four groups. The scores for SNOT-20, CT grade, and endoscopic findings are analyzed in **Supplementary Table 1**.

The article "The Expression of ephrinA1/ephA2 Receptor Increases in Chronic Rhinosinusitis and ephrinA1/ephA2 Signaling Affects Rhinovirus-Induced Innate Immunity in Human Sinonasal Epithelial Cells" was retracted in 2024. Reason: concerns about the images.

### The Expression and Distribution of EphrinA1/ephA2 in Human Sinonasal Mucosa

To determine the role of ephrinA1/ephA2 signaling in human sinonasal mucosa, we surveyed the mRNA transcript levels of ephrin A1 and ephA2 receptor in both sinonasal mucosa and cultured sinonasal epithelial cells. Our results revealed that ephrin A1 and ephA2 receptor are expressed in normal sinonasal mucosa, and their levels were up-regulated in inflammatory sinonasal mucosa of CRS patients, regardless of the existence of nasal polyps. Their levels were not significantly different between patients with CRSsNP and CRSwNP (**Figures 1A-E** and **Supplementary Figure 1**). Consistent with qPCR results, western blot analysis showed upregulated levels of ephrinA1, ephA2 receptor, and phosphorylated ephA2 in inflammatory sinonasal mucosa of patients with CRS compared with those of normal control (**Figures 1B, D** and **Supplementary Figure 1**). Furthermore, the expression levels of ephA2 receptor and phosphorylated ephA2 were also increased in cultured inflammatory epithelial cells, compared with those of normal epithelial cells (**Figure 1E** and **Supplementary Figure 1**). To verify the results of the mRNA and protein analysis, immunofluorescence analysis conducted on section of normal and inflammatory sinonasal mucosal tissues showed the presence of ephA2 in the epithelial and endothelial cells (**Figure 1F**). In addition, ephrinA1 was distributed in the epithelial cells of normal sinonasal mucosa. However, in the inflammatory sinonasal mucosa of patients with CRS, ephrinA1 was found in infiltrating inflammatory cells as well as resident cells such as epithelial cells (**Figure 1F**). Specificity of immunofluorescence staining was verified by neutralization experiments (**Figure 1F**).

**Figure 1:** The expression levels of ephrinA1 (ephA1: **A**, **B**), ephA2 receptor (ephA2: **C, D**), and phosphorylated ephA2 (p ephA2: **D**) in normal and inflammatory sinus mucosa obtained from normal controls (NE, n=25) and patients with CRSsNP (sP, n=36), non-eosinophilic CRSwNP (ncP, n=35), and eosinophilic CRSwNP (ecP, n=38), which were evaluated with real time PCR **(A, C)** and western blots **(B, D)**. **(E)** The expression levels of ephA2 and phosphorylated ephA2 (p ephA2) in cultured epithelial cells derived from normal controls (NE, n=7) and patients with CRSsNP (sP, n=7), non-eosinophilic CRSwNP (ncP, n=7), and eosinophilic CRSwNP (ecP, n=7). Data derived from seven different subjects are presented as dot plots showing median levels. (* means P< 0.05). Upper panels located in Figure **(B, D, E)** show representative protein bands evaluated with western blot. **(F)** The distribution of ephrinA1 (a, c, e, and g) and ephA2 receptor (i, k, m, and o) in normal sinus mucosa (NE; a, i), inflammatory sinus mucosa of patients with CRSsNP (sP: c, k), non-eosinophilic CRSwNP (ncP: e, m), and eosinophilic CRSwNP (ecP: g, o). The results using immunogen for ephrinA1 (b, d, f, and h) and ephA2 receptor (j, l, n, and p) show the disappearance of localization. Large arrow indicates superficial epithelial cells; small arrow indicates blood vessels; arrow heads indicates inflammatory cells. Original magnification x 200.

The article "The Expression of ephrinA1/ephA2 Receptor Increases in Chronic Rhinosinusitis and ephrinA1/ephA2 Signaling Affects Rhinovirus-Induced Innate Immunity in Human Sinonasal Epithelial Cells" was retracted in 2024. Reason: concerns about the images.

### Type 1 and 2 Cytokines, RV, and Poly (I:C) Enhanced Increased Production of EphrinA1/ephA2

Considering that CRSwNP and CRSsNP are associated with increased expression of ephrinA1 and ephA2 receptor in inflammatory sinonasal mucosa, we sought to determine whether Type 1 and Type 2 cytokines relevant to CRS participate in the expression levels of ephrinA1 and ephA2 receptors. Expression of ephrinA1 and ephA2 receptor mRNA levels was also noted in cultured epithelial cells, indicating that these proteins are localized in superficial epithelial cells of sinonasal mucosa (**Figures 1E, F**). As shown in **Figure 2**, the levels of both ephrinA1 and the ephA2 receptor increased in cells treated with TNF-α, IFN-γ, IL-4, IL-5, and IL-13 compared with those of the control group (**Figures 2A, C** and **Supplementary Figure 2**). The levels of both molecules were also similarly upregulated in cultured normal and inflammatory epithelial cells exposed to RV and poly(I:C) (**Figures 2B, D** and **Supplementary Figures 2**, **3**). Furthermore, the level of phosphorylated ephA2 receptor was also significantly upregulated in these cells, indicating that the ephA2 receptor is activated upon stimulation with Type 1 and Type 2 cytokines, poly (I:C), and RV (**Figures 2C**–**E** and **Supplementary Figures 2**, **3**).

**Figure 2:** The expression levels of ephrin A1 **(A)**, ephA2 **(C)**, and phosphorylated ephA2 **(C)** in cultured normal epithelial cells treated with cytokines **(A, C)** at a concentration of 10 ng/ml for 24 h. The expression levels of ephrin A1 **(B)**, ephA2(D), and phosphorylated ephA2 **(E)** in cultured normal (NE) and inflammatory epithelial cells (sP, ncP, and ecP) stimulated with poly (I:C) (10 ng/ml) and rhinovirus for 24 h. Upper panels located in figure **(A–D)** show representative protein bands evaluated with western blot. Data derived from seven different subjects are presented as dot plots showing median levels. (* indicates P< 0.05). Control means non-treated cultured epithelial cells. P ephA2 indicates phosphorylated ephA2. NE, normal epithelial cells; sP; epithelial cells derived from patients with CRSsNP, ncP; epithelial cells derived from patients with neutrophilic CRSNP, ecP; epithelial cells derived from patients with eosinophilic CRSNP.

The article "The Expression of ephrinA1/ephA2 Receptor Increases in Chronic Rhinosinusitis and ephrinA1/ephA2 Signaling Affects Rhinovirus-Induced Innate Immunity in Human Sinonasal Epithelial Cells" was retracted in 2024. Reason: concerns about the images.

### Chemokine Secretion in Sinonasal Epithelial Cells Was Induced by EphrinA1 Treatment

To evaluate the functional effects of ephrinA1 in the sinonasal mucosa, we cultured primary human sinonasal epithelial cells at ALI. First, we investigated whether ephrinA1 regulates the secretion of chemokines in the sinonasal mucosa by stimulating cells with ephrinA1 at 1, 10, 25, and 50 ng/ml doses. The production of chemokines, including IL-8, significantly increased in cells stimulated with ephrinA1 as compared with that in the control, or scrambled siRNA. The production of chemokines was increased in dose- and time- dependent manner (not shown). To determine whether ephA2 is the receptor responsible for the change in the secretion of chemokines induced by ephrinA1, we repeated these experiments in cells transfected with ephA2 siRNA or treated with ephA2 inhibitor. These treatments attenuated the ephrinA1-induced increase in levels of chemokines, indicating that this upregulation in expression is mediated by the ephA2 receptor (**Figure 3A**).

**Figure 3:** **(A)** The expression levels of chemokines such as IL-8, IL-6, ENA78, MIP1-a, RANTES, and MCP-1 in cells stimulated with ephA1 (10 ng/ml) for 24 h. Blocking of ephA2 with ephA2 siRNA or ephA2 inhibitor ameliorated the secretion of chemokines (IL-8. IL-6, ENA78, MIP1-a. RANTES, and MCP-1) induced by ephrinA1 (10 ng/ml) in cultured epithelial cells. * indicates statistical significance P< 0.05 versus ephrinA1 or scrambled siRNA (scr siRNA) + ephirnA1. **(B, C)** Blocking of ephA2 with ephA2 siRNA or ephA2 inhibitor ameliorated the secretion of chemokines (IL-8. IL-6, ENA78, MIP1-a. RANTES, and MCP-1) enhanced by rhinovirus **(B)** or poly (I:C) for 24 h **(C)**. * indicates statistical significance P< 0.05 versus rhinovirus or poly(I:C) or scrambled siRNA (scr siRNA) + rhinovirus or poly(I:C). All data derived from seven different subjects are presented as dot plots showing median levels. (* indicates P < 0.05)

### RV and Poly(I:C) Enhanced the Secretion of Chemokines in Sinonasal Epithelial Cells *via* EphrinA1/ephA2 Signaling Pathway

After finding that ephA2 levels are increased in inflamed sinonasal mucosa derived from CRS patients and upregulated in epithelial cells infected with RV and stimulated with TLR 3 agonist, poly(I:C), the functional significance of ephA2 receptor signaling was evaluated by analyzing the production of chemokines induced by RV and poly(I:C). Compared with those in the control, the levels of IL-8, IL-6, ENA78, MIP-1a, RANTES, MCP-1 were increased in RV-infected epithelial cells. These effects were attenuated by blocking ephA2 with ephA2 siRNA or ephA2 inhibitor, suggesting that the inflammatory action of RV is also supported by ephA2 receptor (**Figure 3B**). Similar findings were found in cells stimulated with poly(I:C) (**Figure 3C**).

The article "The Expression of ephrinA1/ephA2 Receptor Increases in Chronic Rhinosinusitis and ephrinA1/ephA2 Signaling Affects Rhinovirus-Induced Innate Immunity in Human Sinonasal Epithelial Cells" was retracted in 2024. Reason: concerns about the images.

### EphrinA1 Attenuated the Production of Antiviral Immune Mediators *via* EphA2 Receptor

We next evaluated whether activation of ephA2 by ephrinA1 participates in the production of antiviral immune mediators, including IFNs in the sinonasal mucosa. The mRNA levels of antiviral immune mediators such as type I (IFN-β) and III IFNs (IFN-λ1 and IFN-λ2), and ISGs (viperin, Mx, and OAS) were decreased in cultured cells treated with ephrin A1 (**Figure 4A**). In parallel with the mRNA data, the levels of type I (IFN-β) and III IFNs (IFN-λ1 and IFN-λ2) analyzed by ELISA and the levels of ISGs analyzed with western blotting were also decreased in cells stimulated with ephrin A1 (**Figures 4B, C** and **Supplementary Figure 4**). However, their levels were restored in cells transfected with ephA2 siRNA or treated with ephA2 inhibitor (**Figure 4**).

**Figure 4:** The expression levels of IFN-β, IFN-λ1, IFN-λ2, viperin, Mx, and OAS mRNA transcripts **(A)** and protein levels (**B**; ELISA and **C**; western blot) in cultured non-treated epithelial cells (cont), in cells treated with ephrinA1 (10 ng/ml), in cells transfected with scrambled siRNA followed by ephrinA1 treatment (scr siRNA+ephrinA1), in cells transfected with ephA2 siRNA followed by ephrin A1 treatedment (ephrin A1 + ephA2 siRNA), in cells treated with ephA2 inhibitor followed by ephrinA1 treatment (ephA2 inhibitor + ephrinA1). Panels located in figure **(C)** show representative protein bands evaluated with western blot. Data derived from seven different subjects are presented as dot plots showing median levels.* indicates statistical significance P < 0.05 versus ephrinA1 or scr siRNA +ephrinA1.

### EphrinA1/ephA2 Signaling Participates the Production of Antiviral Immune Mediators in RV-infected and Poly(I:C)-Treated Cells

Finally, we assessed whether ephrinA1/ephA2 signaling is involved in the expression of antiviral immune mediators in RV-infected cells or poly(I:C)-treated cells. As expected, antiviral immune mediators were increased in cells infected by RV (**Figures 5A**–**C** and **Supplementary Figure 5**) and stimulated with poly(I:C) (**Figures 5D**–**F** and **Supplementary Figure 5**) compared with those in the control. However, the upregulation of these antiviral immune mediators induced by RV or poly (I;C) was attenuated by ephrinA1 pretreatment (**Figure 5**). When cells transfected with ephA2 siRNA or treated with ephA2 inhibitor were subsequently followed by RV infection or poly(I:C) treatment, the levels of antiviral immune mediators were more upregulated in comparison to those in cells stimulated only with either RV-infection or poly(I:C) alone (**Figure 5**). These results suggest that the ephrinA1/ephA2 signaling dampens epithelial production of type I and type III IFNs, and ISGs enhanced by RV infection or poly (I:C) treatment (**Figure 5**).

The article "The Expression of ephrinA1/ephA2 Receptor Increases in Chronic Rhinosinusitis and ephrinA1/ephA2 Signaling Affects Rhinovirus-Induced Innate Immunity in Human Sinonasal Epithelial Cells" was retracted in 2024. Reason: concerns about the images.

**Figure 5:** **(A–C)** The expression levels of IFN-β, IFN-λ1, IFN-λ2, viperin, Mx, and OAS evaluated by real time PCR **(A, D)**, ELISA **(B, E)**, and western blot **(C, F)** in non-treated epithelial cells (^^; cont), in epithelial cells stimulated with rhinovirus (▪), in ephrinA1-pretreated cells followed by rhinoviral infection (♦; ephrinA1 + rhinovirus), in cells transfected with scr siRNA followed by rhinovirus infection (▲scr siRNA + rhinovirus), in cells transfected with ephA2 siRNA followed by rhinovirus infection (●ephA2 siRNA + rhinovirus), and in cells treated with ephA2 inhibitor followed by rhinovirus infection (^^ephA2 inhibitor + rhinovirus). * denotes statistical significance p < 0.05 versus control, ephrinA1+rhinovirus, ephA2 siRNA + rhinovirus, and ephA2 inhibitor + rhinovirus. ** denotes statistical significance p < 0.05 versus control, rhinovirus, scr siRNA + rhinovirus, ephA2 siRNA + rhinovirus, and ephA2 inhibitor + rhinovirus. # denotes statistical significance p < 0.05 versus control, rhinovirus, ephrinA1+rhinovirus, and scr siRNA+ rhinovirus. **(D–F)**; The expression levels of IFN-β, IFN-λ1, IFN-λ2, viperin, Mx, and OAS evaluated by real time PCR **(A, D)**, ELISA **(B, E)**, and western blot **(C, F)** in non-treated epithelial cells (^^; cont), in epithelial cells stimulated with poly(I:C) (▪), in ephrinA1-pretreated cells followed by poly(I:C) treatment [♦; ephrinA1 + poly(I:C)], in cells transfected with scr siRNA followed by poly(I:C) treatment [▲; scr siRNA + poly(I:C)], in cells transfected with ephA2 siRNA followed by poly(I:C) treatment (●; ephA2 siRNA + poly(I:C)), and in cells treated with ephA2 inhibitor followed by poly(I:C) treatment [??? ephA2 inhibitor + poly(I:C)]. Upper panels located in figure **(C, F)** show representative protein bands evaluated with western blot. All data from seven different subjects are presented as dot plots showing median levels. (P < 0.05). * denotes statistical significance p < 0.05 versus control, ephrinA1+poly(I:C), ephA2 siRNA + poly(I:C), and ephA2 inhibitor + poly(I:C). ** denotes statistical significance p < 0.05 versus control, poly(I:C), scr siRNA + poly(I:C), scr siRNA + poly(I:C), and ephA2 inhibitor + poly(I:C). # denotes statistical significance p < 0.05 versus control, poly(I:C), ephrinA1+ poly(I:C), and scr siRNA+ poly(I:C).

The article "The Expression of ephrinA1/ephA2 Receptor Increases in Chronic Rhinosinusitis and ephrinA1/ephA2 Signaling Affects Rhinovirus-Induced Innate Immunity in Human Sinonasal Epithelial Cells" was retracted in 2024. Reason: concerns about the images.

### The EphrinA1/ephA2 Signaling Enhanced the Phosphorylation of PI3K-Akt-NF-κB and Attenuated the Phosphorylation of TBK/IKKϵ/IRF3

Given that the protective effect of ephA2 blocking in RV-induced inflammation, we investigated whether the ephrinA1/ephA2 signaling would affect the existing signaling pathways; PI3K-Akt-NF-κB pathway leading to the activation of host innate immune genes such as chemokines and TBK/IKKϵ/IRF3 pathway utilized in the secretion of antiviral immune mediators including IFNs and ISGs (12, 14, 42). The levels of proteins in PI3K-Akt-NF-κB and TBK/IKKϵ/IRF3 pathway in cells stimulated with ephrinA1, RV, and poly (I:C) were assessed by western blot analysis. The data demonstrated that phosphorylation of PI3K, Akt, and NF-κB p65 was significantly enhanced by RV infection, poly(I:C), or ephrinA1 treatment, but not in cells transfected with ephA2 siRNA or treated with ephA2 inhibitor (**Figure 6** and **Supplementary Figures 6**, **7**). The phosphorylation of TBK/IKKϵ/IRF3 was enhanced upon exposure to RV and poly(I:C) (**Figure 7** and **Supplementary Figure 8**). However, the phosphorylation of TBK/IKKϵ/IRF3 enhanced by rhinovirus or poly (I:C) was attenuated in cells pretreated with ephrin A1 (**Figures 7A, B** and **Supplementary Figure 8**). Blocking of ephA2 results in more increased phosphorylation of TBK/IKKϵ/IRF3 compared with that in cells stimulated only with either RV or poly(I:C) (**Figures 7C, D** and **Supplementary Figure 9**). These data suggest that ephrinA1/ephA2 signaling may be involved in RV-induced activation of downstream signaling pathways, such as the PI3K/Akt/NF-κB and TBK/IKKϵ/IRF3 signaling pathways. In addition, the inhibition of the TBK/IKKϵ/IRF3 phosphorylation resulted in the decreased expression of antiviral immune mediators including IFN and ISGs, confirming that TBK/IKKϵ/IRF3 pathway participate in the secretion of antiviral immune mediators (**Figure 8**, **9** and **Supplementary Figure 10**).

**Figure 6:** The expression levels of PI3K, phosphorylated PI3K, Akt, and phosphorylated Akt in non-treated epithelial cells (cont), in epithelial cells treated with ephrinA1 (**A**; 10 ng/ml), rhinoviral infection **(B)**, and poly (I:C) **(C)**, and in cells transfected with scrambled siRNA (scr siRNA), ephA2 siRNA, and treated with ephA2 inhibitor followed by ephrinA1 treatment **(A)**, rhinoviral infection **(B)**, and poly(I:C) treatment **(C)**. The expression levels of NF-kB and phosphorylated NF-kB in non-treated epithelial cells (cont), in cells treated with ephrinA1 treatment **(D)**, rhinoviral infection **(E)**, and poly (I:C) treatment **(F)**, and in epithelial cells transfected with scr siRNA, ephA2 siRNA, treated with ephA2 inhibitor followed by ephrinA1 treatment **(D)**, rhinoviral infection **(E)**, and poly (I:C) treatment **(F)**. Upper panels located in each figure show representative protein bands evaluated with western blot. All data derived from seven different subjects are presented as dot plots showing median levels. (* indicates P < 0.05).

The article "The Expression of ephrinA1/ephA2 Receptor Increases in Chronic Rhinosinusitis and ephrinA1/ephA2 Signaling Affects Rhinovirus-Induced Innate Immunity in Human Sinonasal Epithelial Cells" was retracted in 2024. Reason: concerns about the images.

**Figure 7:** **(A)** The expression levels of TBK, phosphorylated TBK (pTBK), IKKϵ, phosphorylated IKKϵ (pIKKϵ), IRF3, and phosphorylated IRF3 (pIRF3) in non-treated epithelial cells (cont), in epithelial cells treated with ephrinA1 (10 ng/ml), in rhinovirus-infected cells, and in ephrinA1-pretreated cell followed by rhinoviral infection for 24 h. **(B)** The expression levels of TBK, phosphorylated TBK (pTBK), IKKϵ, phosphorylated IKKϵ (pIKKϵ), IRF3, and phosphorylated IRF3 (pIRF3) in non-treated epithelial cells (cont), in epithelial cells treated with ephrinA1 (10 ng/ml), in poly(I:C)-treated cells, and in ephrinA1-pretreated cell followed by poly(I:C) treatment for 24 h. **(C)** The expression levels of TBK, phosphorylated TBK (pTBK), IKKϵ, phosphorylated IKKϵ (pIKKϵ), IRF3, and phosphorylated IRF3 (pIRF3) in non-treated epithelial cells (cont), in rhinovirus-infected cells, and in cells transfected with scr siRNA, transfected with ephA2 siRNA, and treated with ephA2 inhibitor followed by rhinoviral infection. **(D)** The expression levels of TBK, phosphorylated TBK (pTBK), IKKϵ, phosphorylated IKKϵ (pIKKϵ), IRF3, and phosphorylated IRF3 (pIRF3) in non-treated epithelial cells (cont), in poly(I:C)-treated cells, and in cells transfected with scr siRNA, transfected with ephA2 siRNA, and treated with ephA2 inhibitor followed by poly(I:C) treatment. Upper panels located in each figure show representative protein bands evaluated with western blot. All data derived from seven different subjects are presented as dot plots showing median levels. (* indicates P < 0.05).

**Figure 8:** The expression levels of IFN-β, IFN-λ1, IFN-λ2, viperin, Mx, and OAS in MRT67307 (5 uM) or G140 (5 uM)-pretreated epithelial cells followed by rhinovirus **(A, C, E)** or poly(I:C) for 24 h **(B, D, F)** using real time PCR **(A, B)**, ELISA **(C, D)**, and western blot **(E, F)**. * indicates statistical significance P < 0.05 between control and MRT67307 or G140-treated cells. All data derived from seven different subjects are presented as dot plots showing median levels.

**Figure 9:** The hypothetical molecular mechanisms through which ephrinA1/ephA2 signaling affect the development of rhinovirus-induced innate immune response in sinonasal mucosa of CRS patients. Rhinovirus may upregulate the expression levels of ephrinA1/ephA2 receptor on sinonasal epithelial cells. This response enhances phosphorylation of downstream signal pathway proteins including PI3K/Akt/NF-κB but attenuates phosphorylation of TBK/IKKϵ/IRF3 pathways, contributing to chemokine secretion and inhibition of the production of antiviral immune mediators including IFNs.

The article "The Expression of ephrinA1/ephA2 Receptor Increases in Chronic Rhinosinusitis and ephrinA1/ephA2 Signaling Affects Rhinovirus-Induced Innate Immunity in Human Sinonasal Epithelial Cells" was retracted in 2024. Reason: concerns about the images.

### RV Copy Number Was Decreased in Cells Transfected with EphA2 siRNA and Pretreated with EphA2 Inhibitor

RV copy numbers were assessed in cell lysate. In the cells transfected with scr siRNA or untreated control cells, the mean copy number reached 2900/ul and 2500/ul after 12 h incubation. Thereafter, RV copy number decreased at 48 h. As expected, blocking ephA2 receptor lowered RV copy number at 12 and 24 h (**Figure 10**).

**Figure 10:** The effect of ephA2 receptor on the RV replication in cultured cells. RV copy number change in time in cultured untreated epithelial cells (control), scr siRNA- transfected cells, ephA2 siRNA-transfected cells, and ephA2 inhibitor-treated cells. All data derived from seven different subjects are presented as median levels with upper and lower distribution. * and ** denote statistical significance p < 0.05 versus control (cont) and scr siRNA-transfected cells in time 0 and 6 hr. # and ## denote statistical significance p < 0.05 versus ephA2 siRNA-transfected cells (ephA2 siRNA) and ephA2 inhibitor treated cells (ephA2 inhibitor) in time 0 and 6 hr.

## Discussion

Deficient production of antiviral immune mediators is regarded as an important factor in the RV-induced exacerbation of respiratory diseases, such as asthma, COPD, and CRS (12, 16, 18, 19). Therefore, it is important to clarify the underlying mechanisms leading to these issues. This study demonstrates that the expression of both the ephA2 receptor and its principal ligand, ephrinA1, is upregulated in sinonasal mucosa of CRS patients. The expression levels of phosphorylated ephA2 was also increased in inflammatory sinonasal mucosa and cultured inflammatory epithelial cells. Furthermore, ephrinA1/ephA2 expression and phosphorylation of ephA2 were upregulated in Type 1 and Type 2 cytokines-treated, RV-infected, and poly(I:C)-treated cells, which suggests that ephA2 is activated in the sinonasal mucosa of CRS patients and in RV-infected mucosa. Chemokine production enhanced by ephrinA1 treatment, RV infection, and poly(I:C) treatment was attenuated by blockage of ephA2 activation. More importantly, the production of type I and III IFN and ISGs enhanced by poly (I:C) treatment and RV infection was increased in ephA2 deficient cells, whereas their production was suppressed by ephrin A1 pretreatment. Taken together, our data suggest that ephrinA1/ephA2 signaling may affect the innate antiviral immune response in sinonasal epithelium, providing a cellular mechanism for RV-induced development and exacerbations of CRS.

The article "The Expression of ephrinA1/ephA2 Receptor Increases in Chronic Rhinosinusitis and ephrinA1/ephA2 Signaling Affects Rhinovirus-Induced Innate Immunity in Human Sinonasal Epithelial Cells" was retracted in 2024. Reason: concerns about the images.

Upregulation of ephrinA1 and ephA2 in CRS patient is consistent with their upregulation, which has been reported in a variety of inflammatory diseases such as pulmonary inflammation and inflammatory bowel disease (30, 31, 43, 44). Epidermal ephA2 expression is upregulated in keratinocytes by several pro-inflammatory cytokines, growth factors, and ultraviolet radiation (45). Hypoxia upregulates both molecules in the skin and lung (29, 46). In endothelial cells, proinflammatory cytokines including TNF-α and IL-1β induced the expression of ephrinA1/ephA2 (47). Exposure of tobacco smoke and lipopolysaccharides in the lung and intestine upregulates the expression of ephrinA1/ephA2 in epithelial cells, pneumocytes, and alveolar macrophages (30–32). In the present study, the levels of ephrinA1/ephA2 are upregulated by CRS-relevant Type 1 and Type 2 cytokines, RV infection, and poly(I:C). Furthermore, the phosphorylated level of ephA2, indicating the activation of ephA2, was also increased in cells exposed to cytokines, RV, and poly(I:C) and was increased in inflammatory sinonasal mucosa and epithelial cells derived from CRS patients. Given that activation of ephA2 is phosphorylation-dependent (48), the present study indicates that the ephrinA1/ephA2 signaling is activated in inflamed sinonasal mucosa of CRS patients, suggesting the possibility that ephrinA1/ephA2 signaling plays a crucial role in RV-induced exacerbations of CRS.

In this study, chemokine production induced by ephrinA1 was attenuated in cells transfected with ephA2 siRNA or treated with ephA2 inhibitor. These findings suggest that ephrinA1 ligand may generate chemokines through the action of ephA2 receptor in sinonasal mucosa. These suggestions are supported by results showing that ligand stimulation by ephrinA1 in pulmonary endothelial cells triggers the expression of CXCL1 and CCL2 but not in endothelial cells treated with ephA2 siRNA (30). Similar results were obtained in LPS-injured lung injury, where the expression of IL-6 and TNF-α decreased in lung tissue of mice with ephA2 mAb pretreatment (30). Furthermore, RV infection or poly (I:C) treatment enhanced the secretion of chemokines in sinonasal epithelial cells, which was also attenuated by blocking the action of ephA2 with ephA2 siRNA or receptor antagonist. On the other hand, the PI3K/Akt pathway lead to the activation of host innate immune genes such as chemokines (42). In parallel with these results, our results showed that the phosphorylation of PI3k/Akt/NF-κB pathway proteins was increased in cells exposed to ephrinA1, RV infection, and poly(I:C). Their phosphorylation was suppressed by blocking ephA2 action, demonstrating that antagonizing ephA2 action may block the PI3k/Akt/NF-κB pathway. These data support the previous study that ephA2 antagonism blocks PI3k/Akt/NF-κB pathway in lipopolysaccharide-induced lung injury (30). Taken together, these results suggest that RV infection or an TLR3 stimulation may contribute to produce chemokines in sinonasal epithelial cells through the ephA2 receptor, activating PI3k/Akt/NF-κB pathway.

The article "The Expression of ephrinA1/ephA2 Receptor Increases in Chronic Rhinosinusitis and ephrinA1/ephA2 Signaling Affects Rhinovirus-Induced Innate Immunity in Human Sinonasal Epithelial Cells" was retracted in 2024. Reason: concerns about the images.

The important aspect of host defense during viral infection is the release of chemokines in the respiratory epithelial cells that leads to an influx of neutrophils, lymphocytes, and eosinophils into the airways (49). An influx of these cells needs to occur in the respiratory mucosa to eliminate viral infection. In this respect, blocking of ephA2 receptor could have harmful influences in the airways, suppressing antiviral host defense. In contrast, these inflammatory responses are implicated in viral exacerbations of asthma and COPD through the secretion of various inflammatory mediators (15–20). Indeed, the combination of RV infection and TNF-α, a cytokine increased in the airway mucosa of patients with asthma and COPD, significantly increased IL-8, ENA78, and GM-CSF in epithelial cells (50). These data suggest that RV infection may aggravate preexisting inflammatory reaction of airway mucosa through chemokine secretion, providing a cellular mechanism leading to RV-induced exacerbations of airway disease. Furthermore, upregulated levels of IL-8 were noted in nasal lavage fluid obtained from asthmatic patients after RV infection, in contrast to levels found in healthy individual (51). Our previous studies showed that chemokines, including CXCL1, CXCL2, and IL-8, were upregulated in cultured epithelial cells obtained from patients with CRS (52). In this respect, blocking ephA2 receptor could provide protective influences in the airway, suppressing unwanted inflammatory responses. These conflicting results require further studies on the role of ephA2 in the sinonasal mucosa of patients with CRS.

Activation of TLR3 induces secretion of IFNs and expression of ISGs to combat the viral infection (53). These concepts are supported by our current data showing that the secretion of antiviral immune mediators including IFN and ISGs are increased in cells stimulated with RV or TLR3 agonist. In contrast to the effect of RV-infection and TLR agonists on the chemokine secretion, which was attenuated by blocking the action of ephA2, we found that the secretion of IFNs and expression of ISGs were more increased rather than been suppressed in cells pretreated with ephA2 siRNA or ephA2 inhibitor. However, the precise molecular mechanism by which the secretion of antiviral immune mediators is increased by blocking the ephA2 receptor are not fully understood. We observed that the secretion of antiviral immune mediators was decreased in cells treated with ephrinA1, which was restored by blocking the ephA2 receptor, compared to those of non-treated epithelial cells. Furthermore, ephrinA1-pretreated epithelial cells followed by rhinovirus infection or poly(I:C) treatment showed decreased expression of antiviral immune mediators, compared to those of cells treated with rhinoviral infection or poly(I:C) treatment alone. These data led us to postulate that basal secretion of ephrinA1 in epithelial cells may results in decreased secretion of antiviral immune mediators through ephA2 receptor. Furthermore, the levels of ephrinA1, ephA2 receptor, and phosphorylated form of ephA2 were increased in inflammatory sinonasal mucosa and their levels were up-regulated in cells treated with RV-infection and poly(I:C). Based on these data, the present study suggests the possibility that the secretion of antiviral immune mediators induced by RV-infection and poly(I:C) may be more increased by inhibiting the action of ephA1 through the blockage of ephA2 receptor.

The article "The Expression of ephrinA1/ephA2 Receptor Increases in Chronic Rhinosinusitis and ephrinA1/ephA2 Signaling Affects Rhinovirus-Induced Innate Immunity in Human Sinonasal Epithelial Cells" was retracted in 2024. Reason: concerns about the images.

Viral infection of respiratory epithelial cells activates a number of signaling cascades including tank binding kinase 1 (TBK1), inhibitor-kB kinase ϵ (Ikkϵ), and IRF3, resulting in the secretion of effector molecules including IFNs and ISGs to induce an antiviral state (12, 14, 54, 55). In the present study, the inhibition of TBK1/Ikkϵ/IRF3 pathway also resulted in decreased secretion of antiviral immune mediators including IFNs and ISGs in sinonasal epithelial cells. However, little is known about crosstalk between signaling cascades, including TBK/IKKϵ/IRF3 and ephA2 receptor in epithelial cells of sinonasal mucosa. In the present study, TBK/IKKϵ/IRF3 phosphorylation was enhanced in cells infected with RV or treated with poly(I:C), but not in cells treated with ephrinA1. Furthermore, TBK/IKKϵ/IRF3 phosphorylation was not induced in ephrinA1-pretreated cells followed by RV infection or poly(I:C) treatment. As well, TBK/IKKϵ/IRF3 phosphorylation induced by RV or poly(I:C) exposure was upregulated by blocking the action of ephA2 compared to those of cells stimulated with RV or poly(I:C) alone. Therefore, our findings have revealed a previously unknown regulatory mechanism between TBK/IKKϵ/IRF3 phosphorylation and ephA2 receptor. Based on these results, we suggest that the inhibition of TBK/IKKϵ/IRF3 phosphorylation by ephrinA1 may contribute to the inactivation of these pathways, resulting in decreased secretion of antiviral immune mediators. In parallel with these findings, TBK/IKKϵ/IRF3 phosphorylation induced by RV-infection and poly(I:C) may be more increased by inhibiting the action of ephA1 through the blockage of ephA2 receptor. These suggestions are supported by the results that the secretion of antiviral immune mediators is attenuated in cells treated with ephrinA1 and is up-regulated in cells transfected with ephA2 siRNA or treated with ephA2 inhibitor. In addition, the present results showed that blocking ephA2 receptor decreases RV replication. Considering the evidences that ephA2 receptor is a functional entry receptor for microbial organisms (24, 25), ephA2 receptor may act as an entry receptor for RV in the sinonasal mucosa, modulating antiviral innate immune response.

The article "The Expression of ephrinA1/ephA2 Receptor Increases in Chronic Rhinosinusitis and ephrinA1/ephA2 Signaling Affects Rhinovirus-Induced Innate Immunity in Human Sinonasal Epithelial Cells" was retracted in 2024. Reason: concerns about the images.

In conclusion, ephrinA1/ephA2 are expressed in normal sinonasal mucosa and their levels are upregulated in inflamed sinonasal mucosa of patients with CRS. RV infection-induced chemokine secretion was ameliorated by blocking ephA2 receptor. Unexpectedly, the production of antiviral immune mediators, including type I and type III IFNs, was increased by blocking ephA2. These results suggest that the ephrinA1/ephA2 signaling may contribute to the innate antiviral immune response in the sinonasal mucosa, providing new therapeutic targets for the management of CRS development and exacerbation.

## Data Availability Statement

The original contributions presented in the study are included in the article/**Supplementary Material**. Further inquiries can be directed to the corresponding author.

## Ethics Statement

The studies involving human participants were reviewed and approved by the review board and ethics committee of Korea University Hospital. The patients/participants provided their written informed consent to participate in this study.

## Author Contributions

SHL conceived and designed the study and performed experiments. SHK, MSH, JWK, and HGK performed the enrollment of patients, collection of samples, and experiments and analyzed data. THL, DBL, and THK performed the enrollment of patients, collection of samples, and experiments, analyzed data and contributed to data visualization. All authors contributed to the article and approved the submitted version.

## Funding

This work was supported by The Basic Science Research Program through the National Research Foundation of Korea (2019R1F1A1058697).

The article "The Expression of ephrinA1/ephA2 Receptor Increases in Chronic Rhinosinusitis and ephrinA1/ephA2 Signaling Affects Rhinovirus-Induced Innate Immunity in Human Sinonasal Epithelial Cells" was retracted in 2024. Reason: concerns about the images.

## Conflict of Interest

The authors declare that the research was conducted in the absence of any commercial or financial relationships that could be construed as a potential conflict of interest.

## Publisher’s Note

All claims expressed in this article are solely those of the authors and do not necessarily represent those of their affiliated organizations, or those of the publisher, the editors and the reviewers. Any product that may be evaluated in this article, or claim that may be made by its manufacturer, is not guaranteed or endorsed by the publisher.

## Supplementary Material

Supplementary Figure 1 Western blot images of **Figures 1B, D, E** including markers.

Supplementary Figure 2 Western blot images of **Figures 2A, B** including markers.

Supplementary Figure 3 Western blot images of **Figures 2C, D** including markers.

Supplementary Figure 4 Western blot images of **Figure 4C** including markers.

Supplementary Figure 5 Western blot images of **Figures 5C, F** including markers.

Supplementary Figure 6 Western blot images of **Figures 6A**–**C** including markers.

Supplementary Figure 7 Western blot images of **Figures 6C**–**F** including markers.

Supplementary Figure 8 Western blot images of **Figures 7A, B** including markers.

Supplementary Figure 9 Western blot images of **Figures 7C, D** including markers.

Supplementary Figure 10 Western blot images of **Figures 7D**, **8E, F** including markers.
